# Research on DNA-Binding Protein Identification Method Based on LSTM-CNN Feature Fusion

**DOI:** 10.1155/2022/9705275

**Published:** 2022-06-02

**Authors:** Weizhong Lu, Xiaoyi Chen, Yu Zhang, Hongjie Wu, Yijie Ding, Jiawei Shen, Shixuan Guan, Haiou Li

**Affiliations:** ^1^School of Electronic and Information Engineering, Suzhou University of Science and Technology, Suzhou 215009, China; ^2^Provincial Key Laboratory for Computer Information Processing Technology, Soochow University, China; ^3^Suzhou Industrial Park Institute of Services Outsourcing, Suzhou 215123, China; ^4^Yangtze Delta Region Institute (Quzhou), University of Electronic Science and Technology of China, Quzhou, 324000, P.R, China

## Abstract

Protein is closely related to life activities. As a kind of protein, DNA-binding protein plays an irreplaceable role in life activities. Therefore, it is very important to study DNA-binding protein, which is a subject worthy of study. Although traditional biotechnology has high precision, its cost and efficiency are increasingly unable to meet the needs of modern society. Machine learning methods can make up for the deficiencies of biological experimental techniques to a certain extent, but they are not as simple and fast as deep learning for data processing. In this paper, a deep learning framework based on parallel long and short-term memory(LSTM) and convolutional neural networks(CNN) was proposed to identify DNA-binding protein. This model can not only further extract the information and features of protein sequences, but also the features of evolutionary information. Finally, the two features are combined for training and testing. On the PDB2272 dataset, compared with PDBP_Fusion model, Accuracy(ACC) and Matthew's Correlation Coefficient (MCC) increased by 3.82% and 7.98% respectively. The experimental results of this model have certain advantages.

## 1. Introduction

Protein is the most important component in the organism. It is closely related to life activities. As a special protein, DNA-binding protein can interact and bind with DNA to form different structures and functions [1]. The interaction between the protein and DNA is an important basis for cell life activities, which not only can achieve multiple functions such as DNA transcription and replication, but also it has a key role in the regulation of organisms. Therefore, the subject of DNA-binding protein [2] prediction is particularly significant. The prediction of DNA-binding protein is to judge whether a protein can combine with DNA. At present, in accordance with different feature information, the prediction of DNA-binding protein can be split into two categories, one is the method relied on protein structure feature information, and the other is the method relied on protein sequence feature information. Generally, methods relied on protein structure feature information have superior prediction results.

However, the traditional biometric technologies, such as filter combination analysis, X-ray diffraction and other methods, have gradually lagged behind the needs of modern society. Although the prediction accuracy rate is high, but they need strict experimental environment and accurate experimental equipment. These methods are high cost and low efficiency. In particular, the number of protein sequences has increased a lot, and these methods are becoming less and less applicable, which limits the research of proteins. Today, due to the cross-age development of computers, more time-saving and labor-saving machine learning methods [3] have come into the sight of researchers. Many researchers used machine learning methods to model based on the existing protein information, and predict the protein. Compared with the traditional biological experiment recognition technology, machine learning method is more efficient, accurate and simple. Cai et al. [4] first developed SVM-Prot based on SVM [5, 6] algorithm. Ma et al. [7] predicted correlations based on random forest algorithm. Gao et al. [8] proposed DBD-Hunter model to judge whether a protein can combine with DNA. Liu et al. [9] made prediction based on the sequence features of PseAAC (Pseudo Amino Acid Composition) combined with the random forest method. Zhao et al. [10] introduced a new volume fraction correction to extract new information from the complex structure of DNA-binding proteins, and further proposed the binding affinity between protein and DNA. Traditional machine learning methods have realized the recognition of DNA-binding protein to a certain extent. However, the effect of deep learning neural network model is better than that of traditional machine learning experiment, which can more effectively extract and train protein features and improve the accuracy of prediction. Alipanahi et al. [11] CNN model was constructed to identify DNA-binding proteins. Qu et al. [12] contributed a fused model of CNN and RNN for identifying DNA-binding proteins. Du et al. [13] proposed a new framework of MsDBPthat uses deep neural networks for learning and classification, which tested 67% accuracy on dataset PDB2272. Chen et al. [14] built a model based on graphical neural network and developed a protein classification predictor.It's accuracy on PDB2272 reached 64.17%. Li et al. [15] first used CNN to extract protein features, and input the features extracted by CNN into LSTM network for prediction, and the accuracy rate on PDB2272 reached 77.77%.

The model proposed in the paperconstructed a deep learning framework based on two neural network models: LSTM and CNN. The function of LSTM wasto extract protein sequence information, and the function of CNN was to extract useful features in evolutionary information. Finally, the extracted information was fused to train, and the result showed that the model improved the accuracy of prediction.

## 2. Materials and Methods

In this part, firstly, the datasets used in the model are introduced. Then, the framework and experimental process proposed in this paper are explained. Finally, the model algorithm in the experiment are displayed.

### 2.1. The Dataset

We acquired the internationally common dataset PDB14189 from Ma, Guo \& Sun (2016) [7] as train dataset, PDB2272 as test dataset. Both datasets are from the collection of DNA-binding protein in the UniProt database [10]. The PDB14189 dataset is divided into 7129 positive sequences and 7060 negative sequences. The PDB2272 is an independent test dataset. In the dataset, it contains 1153 positive sequences and 1119 negative sequences. This dataset is mainly used to test whether this method is improved compared with other methods [16–21]. The sequence similarity in PDB14189 is no more than 40%, and the sequence similarity in PDB2272 is no more than 25%. The number of positive and negative samples in PDB14189 and PDB2272 datasets are shown in Table 1.

### 2.2. Feature Extraction

#### 2.2.1. The Position-Specific Scoring Matrix

The Position-Specific Scoring Matrix (PSSM) [22, 23] can construct the evolutionary information, whichis vital for biological analysis to do some prediction. Therefore, the PSSM has been worked in many relative researches. In this article, PSSM was obtained by searching the non-redundant (NR) database using PSI-BLAST [24]. The iteration and e-values were set to 3 and 0.001,respectively. The PSSM extracted from the protein was represented by an *L*∗*20*dimensional matrix, and the PSSM can be expressed as follow:

(1) $$\begin{array}{c} PSSM=\left[\begin{array}{cccc} P_{1,1} & P_{1,2} & \cdots & P_{1,20}\\ P_{2,1} & P_{2,2} & \cdots & P_{2,20}\\ \vdots & \vdots & \vdots & \vdots \\ P_{L,1} & P_{L,2} & \cdots & P_{L,20} \end{array}\right] \end{array}$$

Where *L* is the number of rows of the PSSM matrix and represents the length of the protein sequence. 20 is the column number of PSSM matrix, representing 20 different amino acid types. The *P_i,j_*represents the conversion rate of amino acid*i*to amino acid *j*. *P_i,j_* is generally a positive integer or a negative integer. When *P_i,j_*is a positive integer and *P_i,j_*is larger, the probability is higher. Conversely, when *P_i,j_* is a negative integer, the smaller the *P_i,j_*, the smaller the probability.

#### 2.2.2. Sequence Encoding

Feature coding is an important work of deep learning. Different datasets have different features. Therefore, it is particularly important to choose an appropriate coding method. Common coding methods are divided into two categories: One-hot coding and Embedding coding. One-hot encoding can digitize any features. Embedding coding is a mapping, it was used to convert discrete variables into continuous variables.

In the dataset used in this paper, the protein sequence is composed of 20 different amino acids, which are represented by 20 different English letters. Several amino acids are arranged together in order to form a protein sequence. The protein sequence can be expressed as *S = S_1_, S_2_,…, S_n_*, where *S_i_*stands for the *i-th* amino acid in sequence. *S_i_* is shown below: Table 2 shows the Dictionary of 20 amino acids.

(2) $$\begin{array}{c} {\text{S}}_{\text{i}}\in \left\{\text{A},\text{R},\text{F},\text{E},\text{H},\text{D},\text{N},\text{C},\text{V},\text{M},\text{Q},\text{G},\text{I},\text{L},\text{K},\text{P},\text{W},\text{Y},\text{S},\text{T}\right\} \end{array}$$

For different amino acids in protein sequence, One-hot encoding is used. When the wrong residue appears in the protein sequence, we use ‘*X'* instead. When a protein sequence of length *L* is used as input and encoded with one-hot, the output is an*20*∗*L*dimensional matrix. For example, for a protein sequence “*S = ANCKYVHIEN*”, it is encoded in one-hot mode. As shown in Figure 1.

### 2.3. Framework of the Model

At present, deep learning neural network has been widely accepted and achieved good results in many industries. This section mainly describes two common deep learning models used to predict whether protein sequences are binding proteins: convolutional neural network (CNN) [25], long-short term memory networks (LSTM) [26] and their fusion models.

### 2.4. Long-Short Term Memory

Recurrent Neural Network (RNN) is a type of artificial neural network. Because the hidden state (*h_t_*) of RNN has short-term memory function, RNN is often used in the classification task with sequence [27] as input, so RNN is used as the basic model for DNA-binding protein classification. However, for a long input sequence, if the derivative of the activation function is too large or too small, the training loss will become too large or too small in the reverse transfer process layer by layer. These two phenomena are called gradient explosion and gradient disappearance, respectively. In order to ensure that the previous input information can still affect the model prediction after a certain time and reduce the influence of gradient disappearance, we use a variant of RNN-LSTM neural network. LSTM neural network adds cell state (*C_t_*) after hidden state to control the change of hidden state. Compared with the hidden state, the change of cell state is relatively slow, which can strengthen the memory function of LSTM to a certain extent.  Figure 2 shows a classic LSTM cell structure.

In the LSTM cell structure shown in Figure 2.In the gate structure of the neuron, the input gate (*i_t_*) receives all the inputs of the node, including the inputs of the upper neuron and the information of the last time point of the node. The forget gate (*f_t_*) determines the information to be lost by this node, and determines the degree of information forgetting by controlling a value from 0 to 1. Neurons themselves need to determine the retention of information and save useful information. Finally, the experimental results are output by the output gate (*o_t_*). Eachgate structure selects a different activation function. The three gate structures and hidden states are calculated as follows:

(3) $$\begin{array}{c} i_{t}=\sigma \left(W_{xi}\left[h_{t-1},x_{t}\right]+b_{xi}\right)\\ o_{t}=\sigma \left(W_{xo}\left[h_{t-1},x_{t}\right]+b_{xo}\right)\\ f_{t}=\sigma \left(W_{xf}\left[h_{t-1},x_{t}\right]+b_{xf}\right)\\ C_{t}=f_{t}C_{t-1}+i_{t}\tanh\left(W_{xc}\left[h_{t-1},x_{t}\right]+b_{xc}\right)\\ h_{t}=o_{t}\tanh\left(C_{t}\right) \end{array}$$

The specific structure of LSTM can be explained by the above formula. Where the *σ*is the sigmoid function. *i_t_,f_t_,o_t_* are three gate structures of LSTM, respectively. *b* is bias,and *C* is long-term memory in LSTM. *W_xi_, W_xo_,W_xc_* are three corresponding weight matrices of three different gate structures in the LSTM.

### 2.5. Convolutional Neural Network

Convolutional neural network has a very important position in deep learning. Compared with other classification algorithms, convolutional neural network needs much less data processing. In the early machine learning algorithms, the filter of the model was designed manually. However, CNN can learn the data features after enough training. In recent years, many network models have been developed based on convolutional neural networks, mainly including AlexNet [28], VGGNet [29] and ResNet [30].

As shown in Figure 3, Convolutional neural network is usually composed of multi-layer convolution layer and pooling layer. The input data to the model is usually a two-dimensional matrix. Multiple convolution cores are defined and applied to the whole data for convolution process. Finally, the feature mapping matrix corresponding to the convolution core is obtained. Each convolution core represents a feature detector and scans the corresponding features on the data. The pool stage is usually connected behind the convolution layer to reduce the dimension of the feature map by taking the maximum or average value. Deep learning models can usually contain multiple convolution layers to learn more complex abstract features.

### 2.6. Model Fusion

This section mainly displays the deep learning model proposed. As shown in Figure 4, the biggest difference between our proposed model and other existing models is that our model is a parallel structure. LSTM and CNN canextract different information features at the same time. Finally, the extracted information was fused as the input of MultiLayer Perceptron (MLP) [31] for training and classification. Other existing models are series structure, which connects CNN and LSTM in series. In series structure, those two networks cannot extract features at the same time.

The output of the model was a probability value and 0.5 was set as the dividing point. When the output is greater than 0.5, it is predicted that this protein can bind to DNA. When the output is less than 0.5, the result is just the opposite.

### 2.7. Model Algorithm

In this section, the specific algorithm of the model is described in detail. The protein sequence features and PSSM matrix wereput into two parallel neural networks. Finally, the extracted information was fused as the input of MLP full connection layer for training and classification. The specific pseudo algorithm is shown in Algorithm 1.

## 3. Results and Discussion

### 3.1. Evaluation Index

In this experiment, four evaluation indicators were used. They are accuracy (*ACC*), sensitivity (*Sen*), specificity (*Spe*) [32] and Matthew's Correlation Coefficient (*MCC*). The formulas of these four evaluation indexes are as follows:

(4) $$\begin{array}{c} ACC=\frac{\left(TP+TN\right)}{\left(TP+TN+FP+FN\right)}\\ Sen=\frac{TP}{\left(TP+FN\right)}\\ Spe=\frac{TN}{\left(TN+FP\right)}\\ MCC=\frac{\left(TP\times TN\right)-\left(FP\times FN\right)}{\left(\sqrt{\left(TP+FN\right)\times \left(TN+FP\right)\times \left(TP+FP\right)\times \left(TN+FN\right)}\right)} \end{array}$$

*TP* is the size of positive sequences correctly identified.

*TN* is the size of negative sequences correctly identified.

*FP* is the size of negative sequences incorrectly identified.

*FN* is the size of positive sequences incorrectly identified.

*Sen* is sensitivity, which is the percentage of correctly identified positive sequence.

*Spe*is specificity, which is the percentage of correctly identified negative sequence.

*ACC* is accuracy, which is the percentage of correctly identified sequence.

*MCC* is Matthew's Correlation Coefficient, which means the prediction quality of the binary classification model, with a range of [-1,1]. The smaller the *MCC*, the worse the prediction quality of the algorithm [32, 33].

### 3.2. Model Hyperparameter

The experimental code of model in the paper was implemented through the PyTorch framework. In addition, hyperparameters are very important to the model. Only by constantly adjusting the hyperparameters can we get the optimal training model. Hyperparameters are often initially set based on experience. The settings of parameters are shown in Table 3.

### 3.3. Result

In this section, we first compared the comparative experiments based on different length sequences. Next, we considered whether to add a Dropout [34] layer and Regularization, and conducted two sets of comparative experiments. Then, other parameters were selected to obtain the best training model. Finally, wetested on the train dataset PDB14189 and the test dataset PDB2272, and compared the performance with other existing models.

### 3.4. Result of Different Sequence Lengths

In the data processing phase, we select different maximum lengths (from 100 to 900) to encode DNA sequences to evaluate the overall performance.  Figure 5 shows that the result is the best when the protein sequence length is 700.

### 3.5. Model Performance whether Selecting Dropout

When the model was used to train the dataset, it was easy to form an over-fitting phenomenon. In order to prevent the problem, a dropout method was proposed. The direct function of dropout is to reduce the number of intermediate features, so as to reduce redundancy and increase the orthogonality between features in each layer. In each training batch, the interaction between hidden layer nodes is reduced by ignoring the general feature detector to improve experimental results. Comparative experiments are shown in Table 4.

### 3.6. Model Performance whether Selecting Regularization

Like dropout, regularization [35, 36] is also a method to prevent the training model from overfitting. We can understand regularization as “constraint”, which is convenient to understand. The more complex the model, the easier it is to overfit. The role of regularization is to correct the problem. Some are in the model design stage, and some are in the model training stage. The purpose is to prevent overfitting. Therefore, we set the hyperparameter of weight_decay, which is a method of weight decay. Weight decay is to subtract a gradient from the gradient of each update. As shown in the formula (5).In this method, a penalty term is added to the model loss function to make the learned model parameters smaller, which is a common method of overfitting. The results were different when the value of weight_decay was different. The experimental results are shown in Table 5.

(5) $$\begin{array}{c} \theta_{t+1}=\left(1-\lambda \right)\theta_{t}-\alpha \nabla f_{t}\left(\theta_{t}\right) \end{array}$$

*θ* is the model parameter vector, ∇*f*_*t*_(*θ*_*t*_) is the gradient of loss function at *t* time, and *α* is the learning rate.

When other parameters are determined, we adjust weight_decay and find that the training result is best when weight_decay =0.01. So during training, we adjust weight_decay to 0.01 to optimize our final training result.

### 3.7. Result Comparison on the Benchmark Dataset

In order to demonstrate the effectiveness of our proposed model. On the benchmark dataset PDB14189, we compared DNABP [7], MsDBP [13], StackDPPred [22], PDBP-CNN [15] and PDBP-Fusion [15]. The DNABP method adopts various sequence features. The specific experiment comparison is shown in Table 6.

For a visual comparison, we show this as a bar graph in Figure 6.

### 3.8. Result Comparison on the Test Dataset

On the PDB2272 dataset, different methods were compared. In Table 7,the ACC of our proposed model is 81.59%, which is 3.82% higher than the ACCof PDBP_Fusion model. From this indicator of MCC, the MCC of our model is 64.63%, which is 7.98% higher than the MCC of PDBP_Fusion. Therefore, the method has certain advantages.

As shown in Figure 7, the method plays a role in identifying DNA-binding protein. In conclusion, our model is effective. It is a reliable deep learning neural network algorithm.

## 4. Conclusions

DNA-binding proteins are essential for the regulation of life activities. And in pharmaceutical engineering, DNA-binding proteins are key components of steroids, antibiotics, and anticancer drugs. Therefore, the identification of DNA-binding proteins is of great significance. In this paper, good recognition performance is achieved by only extracting protein features and combining deep learning algorithm pairs to determine whether related proteins have a preference for interacting with DNA. The main work of this paper is as follows: a DNA-binding protein fusion recognition model based on LSTM and CNN is proposed. In view of the weak ability of traditional protein feature representation, we use LSTM and CNN to extract protein sequence information and local information, respectively, to improve the ability of protein feature representation. By effectively extracting protein sequence features and local features, the modeling ability of protein depth features and the recognition ability of DNA-binding proteins are significantly improved.

Compared with traditional methods at the forefront of this field, the experimental results verify the superiority and stability of the model. In the future, we plan to use different biological features and continue to improve overfitting to further improve the prediction speed and accuracy of the model.

## Figures and Tables

**Figure 1:** One-hot Encoding.

**Figure 2:** Classic LSTM Cell Structure.

**Figure 3:** Convolutional Neural Network Structure.

**Figure 4:** Network Model.

**Figure 5:** Comparative experiment of different sequence lengths. (a) is the result of different sequence lengths in dataset PDB14189. (b) is the result of different sequence lengths in dataset PDB2272.

**Figure 6:** Result Comparison on PDB14189.

**Figure 7:** Result Comparison on PDB2272.

**Algorithm 1:** Pseudo code of the algorithm.

**Table 1:** Introduction to the dataset.

Number \dataset	PDB14189	PDB2272
DBPs	7129	1153
Non-DBPs	7060	1119
Total	14189	2272

**Table 2:** Dictionary of 20 amino acids.

Amino acid	Sequence	Amino acid	Sequence
Alanine	A	Glutamine	Q
Arginine	R	Glycine	G
Phenylalanine	F	Isoleucine	I
Glutamicacid	E	Leucine	L
Histidine	H	Lysine	K
Asparticacid	D	Proline	P
Asparagine	N	Tryptophan	W
Cysteine	C	Tyrosine	Y
Valine	V	Serine	S
Methionine	M	Threonine	T

**Table 3:** Setting of hyperparameters.

Hyperparameter	Setting
Epoch	70
Learning rate	0.001
Batch size	64
Optimizer	Adam
Loss function	Binary cross entropy loss

**Table 4:** Result comparison of whether selecting Dropout.

	ACC(%)	Sen(%)	Spe(%)	MCC(%)
With dropout	*79.83*	*73.59*	91.35	62.06
Without dropout	*79.44*	*74.29*	87.89	60.32

**Table 5:** Result comparison of different weight_decay.

	ACC(%)	Sen(%)	Spe(%)	MCC(%)
weight_decay =0.1	*66.80*	*64.28*	68.22	32.04
weight_decay =0.01	*81.59*	*76.23*	90.23	64.63
weight_decay =0.001	*78.91*	*72.05*	93.00	61.05
weight_decay =0.0001	*76.75*	*69.62*	93.51	57.78

**Table 6:** Result comparison on PDB14189.

Methods	ACC(%)	Sen(%)	Spe(%)	MCC(%)
MsDBP	80.29	80.87	79.72	60.61
PSSM-PP + PHY	82.67	79.95	85.39	65.4
BP ± NBP + PHY	80.40	76.88	83.92	60.9
PSSM	79.62	76.02	83.21	59.4
64 optimal featuresa	86.90	83.76	90.03	72.2
PHY	77.65	73.54	81.76	55.5
PSSM-PP + BP_NBP	83.68	81.01	86.34	67.4
PSSM-PP	81.69	78.92	84.45	63.5
ALL features	84.64	82.23	87.06	70.6
StackDPPred(one-hot)	76.00	79.27	72.71	52.10
PDBP-CNN	82.02	87.49	76.50	64.69
PDBP-fusion	82.81	86.45	79.13	66.1
Our methods	96.93	96.46	97.41	93.86

**Table 7:** Result comparison on PDB2272.

Methods	ACC(%)	Sen(%)	Spe(%)	MCC(%)
Qu et al. [12]	48.33	49.07	48.31	−3.34
DPP-PseAAC [17]	58.10	59.10	56.63	16.25
MsDBP [13]	66.99	66.42	70.69	33.97
Local-DPP [19]	50.57	58.72	8.76	4.564
PseDNA-Pro [37]	61.88	59.90	75.28	24.30
PDBP-Fusion [15]	77.77	73.31	66.85	56.65
Our methods	81.59	76.23	90.23	64.63

## Data Availability

The dataset is available in the references cited.

## References

[1] Nogueira M. S., Koch O. (2019). The development of target-specific machine learning models as scoring functions for docking-based target prediction. *Journal of Chemical Information and Modeling*.

[2] Kaiyang Q. (2019). A review of DNA-binding proteins prediction methods. *Current Bioinformatics*.

[3] Wei L., Liao M., Gao X., Zou Q. (2015). Enhanced protein fold prediction method through a novel feature extraction technique. *IEEE Transactions on Nanobioscience*.

[4] Cai C. Z., Han L. Y., Ji Z. L. (2003). SVM-Prot: web-based support vector machine software for functional classification of a protein from its primary sequence. *Nucleic Acids Research*.

[5] Qian Y., Meng H., Lu W., Liao Z., Ding Y., Wu H. (2022). Identification of DNA-binding proteins via Hypergraph based Laplacian Support Vector Machine. *Current Bioinformatics*.

[6] Zou Y., Ding Y., Peng L., Zou Q. (2021). FTWSVM-SR: DNA-binding proteins identification via fuzzy twin support vector machines on self-representation. *Interdisciplinary Sciences: Computational Life Sciences*.

[7] Ma X., Guo J., Sun X. (2016). DNABP: Identification of DNA-binding proteins based on feature selection using a random forest and predicting binding residues. *PloS One*.

[8] Gao M., Skolnick J. (2008). DBD-hunter: a knowledge-based method for the prediction of DNA–protein interactions. *Nucleic Acids Research*.

[9] Liu B., Wang S., Wang X. (2015). DNA binding protein identification by combining pseudo amino acid composition and profile-based protein representation. *Scientific Reports*.

[10] Zhao H., Yang Y., Zhou Y. (2010). Structure-based prediction of DNA-binding proteins by structural alignment and a volume-fraction corrected DFIRE-based energy function. *Bioinformatics*.

[11] Alipanahi B., Delong A., Weirauch M. T., Frey B. J. (2015). Predicting the sequence specificities of DNA- and RNA-binding proteins by deep learning. *Nature Biotechnology*.

[12] Qu Y. H., Yu H., Gong X. J., Xu J. H., Lee H. S. (2017). On the prediction of DNA-binding proteins only from primary sequences: a deep learning approach. *PLoS One*.

[13] Du X., Diao Y., Liu H., Li S. (2019). MsDBP: exploring DNA-binding proteins by integrating multiscale sequence information via Chou’s five-step rule. *Proteome Research*.

[14] Chen D., Wei L. (2021). A useful tool for the identification of DNA-binding proteins using graph convolutional network. *Current Proteomics*.

[15] Li G., Du X., Li X., Zou L., Zhang G., Wu Z. (2021). Prediction of DNA binding proteins using local features and long-term dependencies with primary sequences based on deep learning. *Peer J*.

[16] Zeng H., Edwards M. D., Liu G., Gifford D. K. (2016). Convolutional neural network architectures for predicting DNA-protein binding. *Bioinformatics*.

[17] Rahman M. S., Shatabda S., Saha S., Kaykobad M., Rahman M. S. (2018). DPP-PseAAC: A DNA-binding protein prediction model using Chou's general PseAAC. *Theoretical Biology*.

[18] Zhang P., Tao L., Zeng X. (2017). A protein network descriptor server and its use in studying protein, disease, metabolic and drug targeted networks. *Briefings in Bioinformatics*.

[19] Wei L., Tang J., Zou Q. (2017). Local-DPP: An improved DNA-binding protein prediction method by exploring local evolutionary information. *Information Sciences*.

[20] Wang Y., Ding Y., Guo F., Wei L., Tang J. (2017). Improved detection of DNA-binding proteins via compression technology on PSSM information. *PLoS One*.

[21] Zou Y., Wu H., Guo X. (2020). MK-FSVM-SVDD: A Multiple Kernel-based Fuzzy SVM Model for Predicting DNA-binding Proteins via Support Vector Data Description. *Current Bioinformatics*.

[22] Lu W., Song Z., Ding Y. (2020). Use Chou’s 5-Step Rule to Predict DNA-Binding Proteins with Evolutionary Information. *BioMed Research International*.

[23] Wei L., Liao M., Gao X., Zou Q. (2015). An improved protein structural classes prediction method by incorporating both sequence and structure information. *IEEE Transactions on Nanobioscience*.

[24] Schaffer A. A., Aravind L., Madden T. L. (2001). Improving the accuracy of PSI-BLAST protein database searches with composition-based statistics and other refinements. *Nucleic Acids Research*.

[25] Chauhan S., Ahmad S. (2020). Enabling full-length evolutionary profiles based deep convolutional neural network for predicting DNA-binding proteins from sequence. *Proteins: Structure, Function, and Bioinformatics*.

[26] Lample G., Ballesteros M., Subramanian S., Kawakami K., Dyer C. (2016). Neural architectures for named entity recognition. https://arxiv.org/abs/1603.01360.

[27] Klaus G., Rupesh K. S., Jan K., Bas R. S., Jürgen S. (2015). LSTM: a search space odyssey. *IEEE Transactions on Neural Networks and Learning Systems*.

[28] Krizhevsky A., Sutskever I., Hinton G. E. (2012). Imagenet classification with deep convolutional neural networks. *Advances in Neural Information Processing Systems*.

[29] Simonyan K., Zisserman A. (2014). Very Deep Convolutional Networks for Large-scale Image Recognition. https://arxiv.org/abs/1409.1556.

[30] He K., Zhang X., Ren S., Sun J. Deep residual learning for image recognition.

[31] Pal S. K., Mitra S. (1992). Multilayer Perceptron, Fuzzy Sets, Classifiaction. *IEEE Transactions on Neural Networks*.

[32] Lu W., Song Z., Ding Y., Wu H., Huang H. A Prediction Method of DNA-Binding Proteins Based on Evolutionary Information.

[33] Wang X.-F., Gao P., Liu Y.-F., Li H.-F., Fan L. (2020). Predicting thermophilic proteins by machine learning. *Current Bioinformatics*.

[34] Ding Y., Yang C., Tang J., Guo F. (2022). Identification of protein-nucleotide binding residues via graph regularized k-local hyperplane distance nearest neighbor model. *Applied Intelligence*.

[35] Girosi F., Jones M., Poggio T. (1995). Regularization theory and neural networks architectures. *Neural Computation*.

[36] Ide H., Kurita T. Improvement of learning for CNN with ReLU activation by sparse regularization.

[37] Liu B., Xu J., Fan S., Xu R., Zhou J., Wang X. (2015). PseDNA-pro: DNA-binding protein identification by combining chou’s PseAAC and physicochemical distance transformation. *Molecular Informatics*.

